# An Empirical Study on the Inequality in Health and Healthcare in China's Medical Reform

**DOI:** 10.1155/2022/5789118

**Published:** 2022-05-26

**Authors:** Jing-wei Li, Feng Jin

**Affiliations:** ^1^School of Insurance and Economics, University of International Business and Economics, Beijing 100029, China; ^2^School of International Trade and Economics, University of International Business and Economics, Beijing 100029, China

## Abstract

To make clear what role the Urban and Rural Residents Basic Medical Insurance (URRBMI) plays in the inequality in health and healthcare, this article combines the time-varying DID method with the concentration index to conduct an empirical study. We find that the URRBMI improves health but expands health inequality among different income groups, with its contribution growing over time. Besides, the URRBMI significantly promotes healthcare utilization, reduces the medical burden, and narrows the gap among different income groups, though this effect is generally downward. These findings help clarify what deserves more attention to enlarge benefits and reduce inequality in this medical reform and provide policy implications for policymakers. Increasing investment in medical resources and constructing the hierarchical medical system and medical treatment combination may make a difference.

## 1. Introduction

Social health insurance effectively provides universal health and healthcare coverage, especially in developing countries [1]. China's central government established the Urban Employees Basic Medical Insurance (UEBMI), the New Cooperative Medical Insurance (NCMS), and the Urban Residents Basic Medical Insurance (URBMI) in 1998, 2003, and 2007, respectively, as the basic medical insurance system. However, just like some other developing countries, such as Vietnam and Colombia [2, 3], China has to face the inequality coexisting with universal healthcare coverage due to the fragmentation of the Basic Medical Insurance System [4]. The fragmentation gives rise to divisions of eligibility and benefits between urban and rural areas, between different regions, and among social groups [5, 6].

To deal with the fragmentation, China's central government and some local governments began to explore “integrating” the UEBMI, NCMS, and URBMI and carry out the medical insurance reform step by step. The URBMI and NCMS are integrated at the first stage because they share more similarities. The medical insurance is called the Urban and Rural Residents Basic Medical Insurance (URRBMI) after the “integrating” reform, and we use the URRBMI to represent the reform in this article.

China's central government issued the “Opinions on Integrating the Basic Medical Insurance Systems for Urban and Rural Residents” (“Opinions” below), including six aspects: integrating the coverage, integrating the fundraising policies, integrating the benefits and reimbursement rates, integrating the drug list, integrating the healthcare providers, and integrating the fund management [7]. Before the Opinions, local governments made spontaneous and initial exploration according to local conditions, which we call the “spontaneous integration” stage. However, the URRBMI progressed slowly in this stage. As shown in Figure 1, only 400 million people participated in the URRBMI before 2016. The Opinions marks that the URRBMI has entered the “full implementation” stage. We can see a sharp increase in the URRBMI's participants since the issue of the Opinions and doubled from 2016 to 2018 in Figure 1.

This study combines the time-varying DID and concentration index. By calculating and decomposing inequality in China based on the panel data from the China Labor-force Dynamic Study (CLDS), we find that: (1) There is “pro-rich” inequality in health and “pro-poor” inequality in healthcare. (2) The URRBMI significantly improves health. But it deepens the “pro-rich” health inequality, with its contribution to health inequality increasing year by year. (3) The URRBMI promotes healthcare utilization, effectively reduces the medical burden, and narrows the gap among different income groups. Its contribution to the “pro-poor” healthcare inequality declines with time. (4) The decomposition results of inequality between groups show that the URRBMI plays a different role in different areas and regions. (5) The lowest-income people benefit the most from the URRBMI.

The rest of this article is organized as follows: Section 2 reviews the existing literature.  Section 3 presents the research methodology.  Section 4 calculates, decomposes, explains, and discusses the inequality in health and healthcare using the CLDS data.  Section 5 concludes and provides policy implications.

## 2. Literature Review

From initial exploration in several places to nationwide promotion, the URRBMI has achieved phased results. Some scholars believe that the URRBMI releases the medical needs of rural residents, promotes the utilization of healthcare services [8, 9], protects health, increases healthcare benefits [10], and receives strong support from the urban and rural residents [11]. In addition, the URRBMI also promotes the access to healthcare and avoids the phenomenon of “the poor help the rich,” which enhances the fairness of the Basic Medical Insurance System [12, 13]. However, some scholars believe that the URRBMI only has a limited effect on healthcare utilization and health outcomes. For example, based on China Health and Retirement Longitudinal Study, Fan et al. find that the URRBMI improves the outpatient healthcare utilization but not the inpatient healthcare utilization [14]. Zhu et al. point out that the financing of the URRBMI is insufficient to meet the demand of people for healthcare and does not significantly narrow the urban-rural gap in fundraising [15]. Focusing on the urban-rural inequality of opportunity, Ma et al. use China Health and Nutrition Survey (CHNS) data to get the fairness gap. Their study shows that the URRBMI fails to eliminate the opportunity gap in healthcare utilization [16]. Moreover, there are considerable differences between areas, regions, and people with different socioeconomic status [17, 18]. Since the URRBMI is a newly implemented medical insurance, the related studies are still not enough and do not reach a consensus conclusion. This study not only adds new empirical evidence on the policy effects of the URRBMI, but also enriches the existing and growing literature that evaluates China's Basic Medical System [19–21].

Some existing studies on the URRBMI mainly treat the URRBMI as a policy shock at a fixed time [12, 16–18]. However, the implementation of the URRBMI varied in time before 2016, the year the Opinions was officially issued. Therefore, the time-varying DID is a better approach to analyze the URRBMI. It can effectively identify the URRBMI's causal effect on health and healthcare. The concentration index is a representative indicator to measure inequality. The decomposition of the concentration index is conducted based on the multiple regression model [10], the difference-in-difference method [12], or the generalized linear mixed model [13]. However, we have not seen studies combining the concentration index with the time-varying DID method. Therefore, this study combines the concentration index with the time-varying DID method to study the URRBMI and inequality. Moreover, this study compares the inequality in health and healthcare both at urban-rural level and region level, trying to make a more comprehensive assessment.

## 3. Research Methodology

### 3.1. Concentration Index and the Decomposition

This study uses the concentration index (CI) to measure the inequality in health and healthcare related to socioeconomic status. Compared with other indicators such as the Lorenz curve, Gini index, etc., CI not only reflects the inequality of the whole population but also highlights the inequality among groups divided by socioeconomic status. We use the income to measure socioeconomic status in this article. The income gap, from the perspective of social policy, is directly related to social welfare and results in income-related inequality in social welfare, such as medical services [22]. Therefore, CI a suitable indicator for our study.  Figure 2 shows the concentration curve as an example. The whole sample is sorted by income, and the income's cumulative percentage is used as the horizontal axis. The vertical axis is the cumulative percentage of the health (or healthcare) variable. It can be called the “Fair Line” if the concentration curve is a straight line of 45 degrees diagonally upward. CI is twice the difference between the area under the Fair Line and the area under the concentration curve, which can be expressed as follows [23, 24]:

(1) $$\begin{array}{c} \text{CI}=1-2\int_{0}^{1}C\left(q\right)\text{d}q, \end{array}$$

where *C*(*q*) denotes the *concentration curve*. The absolute value of CI represents the “size” of the inequality, and the bigger the absolute value of CI, the larger the inequality.

Let *y* be the health or healthcare variable. When *y* is a positive indicator, such as self-rated health status, CI > 0 indicates that the high-income earners have better self-rated health status, which is the “pro-rich” inequality. Moreover, when *y* is a negative indicator, such as out-of-pocket medical expenses,  CI > 0 implies that the high-income earners have a heavier medical burden, which is the “pro-poor” inequality.

The concentration curve and CI can illustrate the existence and the “size” of the inequality. However, if we want to study the specific factors influencing inequality, we need to decompose CI. Assume that *n* factors affect the health or healthcare (*y*), denoted as *x*_*k*_(*k*=1,2,…, *n*), and income is denoted as *I*. According to Wagstaff et al. [25, 26], we decompose the *y*'s CI into the sum of the contributions of all the factors. The contribution of each factor includes two parts: the elasticity of *y* to *x*_*k*_, which means the direct impact on *y*; and the CI of *x*_*k*_, which means the inequality of the factor itself. Therefore, the decomposition can be conducted as follows:

(2) $$\begin{array}{c} \text{CI}\left(y|I\right)=\sum_{k=1}^{n}\eta_{k}\text{CI}\left(x_{k}|I\right)+\frac{{\text{CI}}_{\varepsilon }}{\bar{I}}, \end{array}$$

where *η*_*k*_ is the elasticity of *y* to *x*_*k*_, denoting the percentage of change in *y* caused by every 1% change in *x*_*k*_. That is, the direct impact of *x*_*k*_ on *y*. CI(*x*_*k*_*|I*) is the inequality of *x*_*k*_. Then *η*_*k*_CI(*x*_*k*_*|I*) is the contribution of *x*_*k*_. $\bar{I}$ is the sample mean of *I*; CI_*ε*_ is the CI of the residual term, which represents the unobservable part that cannot be explained by these *n* factors. CI(*x*_*k*_*|I*) can be calculated from the sample data, and *η*_*k*_ requires the regression of each factor *x*_*k*_ against *y* as follows:

(3) $$\begin{array}{c} y=\gamma +\sum_{k=1}^{n}\rho_{k}x_{k}+\varepsilon_{i}. \end{array}$$

*ρ*_*k*_ is the impact of *x*_*k*_ on *y*. Assuming that for each observation, the coefficient vector *ρ*_*k*_ is the same and the individual difference in *y* is only determined by the difference in *x*_*k*_, then we have $\eta_{k}=\rho_{k}\left(\bar{x_{k}}/\bar{y_{k}}\right)$. Therefore, Equation (2) can be further rewritten as follows:

(4) $$\begin{array}{c} \text{CI}\left(y|I\right)=\sum_{k=1}^{n}\rho_{k}\frac{\bar{x_{k}}}{\bar{y_{k}}}\text{CI}\left(x_{k}|I\right)+\frac{{\text{CI}}_{\varepsilon }}{I}. \end{array}$$

To measure the inequality between the urban and rural areas, we divide the sample into urban and rural groups according to where the individual's hukou is located and use this as a standard to decompose the inequality into intragroup inequality and intergroup inequality as follows:

(5) $$\begin{array}{c} \text{CI}\left(y|I\right)=\frac{N_{u}}{N}{\text{CI}}_{u}\left(y|I\right)+\frac{N_{r}}{N}{\text{CI}}_{r}\left(y|I\right)+{\text{CI}}_{ur}\left(y|I\right). \end{array}$$

*N*_*u*_ and *N*_*r*_ represent the sample size of urban and rural residents, and *N* represents the total sample size. CI_*u*_(*y|I*) and CI_*r*_(*y|I*) represent the intragroup inequality of urban and rural residents, respectively, and CI_*ur*_(*y|I*) represents the intergroup inequality between urban and rural areas.

The sample can also be divided into the east and non-east regions in the same way, where the non-east region refers to the middle and west regions. Then, the decomposition of inequality between regions can be written as follows:

(6) $$\begin{array}{c} \text{CI}\left(y|I\right)=\frac{N_{e}}{N}{\text{CI}}_{e}\left(y|I\right)+\frac{N_{ne}}{N}{\text{CI}}_{ne}\left(y|I\right)+{\text{CI}}_{b}\left(y|I\right). \end{array}$$

Similarly, *N*_*e*_ and *N*_*ne*_ represent the sample size in the east and the non-east region, respectively, and CI_*e*_(*y|I*) and *CI*_*ne*_(*y|I*) represent the intragroup inequality of the east and non-east region, respectively. CI_*b*_(*y|I*) is the intergroup inequality between the east and non-east region.

The inequality in health and healthcare changes dynamically over time. To study the roles of different factors, especially the role of the URRBMI, we conduct the Oaxaca decomposition to CI and decompose the dynamic change of inequality into the inequality change of *x*_*k*_ and the change of *y*'s elasticity to *x*_*k*_. It can be expressed as follows:

(7) $$\begin{array}{c} \Delta \text{CI}\left(y|I\right)=\sum_{k=1}^{n}\eta_{kt-1}\Delta \text{CI}\left(x_{k}|I\right)+\sum_{k=1}^{n}{\text{CI}}_{t}\left(x_{k}|I\right)\Delta \eta_{k}. \end{array}$$

CI_*t*−1_(*x*_*k*_*|I*) and *η*_*kt*−1_ represent the CI of *x*_*k*_ and the elasticity of *y* to *x*_*k*_ in the *t*−1 period. The inequality change of *x*_*k*_ is ΔCI(*x*_*k*_*|I*) and the change of *y*'s elasticity to *x*_*k*_ is Δ*η*_*k*_, where ΔCI(*x*_*k*_*|I*)=CI_*t*_(*x*_*k*_*|I*) − CI_*t*−1_(*x*_*k*_*|I*) and Δ*η*_*k*_=*η*_*kt*_ − *η*_*kt*−1_. It can be seen that decomposing the dynamic changes of CI helps clarify the main part of each factor that contributes more to the change of inequality.  Table 1 summarizes the main notations and their definitions in this part.

### 3.2. Data and Variables

The data used in this study are derived from the China Labor-force Dynamic Study (CLDS) organized by the Social Science Survey Center of Sun Yat-sen University, whose baseline survey was conducted in 2012, with follow-up surveys conducted every 2 years. The data cover the labor population aged 15 to 64 in 29 provinces, autonomous regions, and municipalities in China and contains vast amounts of comprehensive and high-quality information, such as health status, income, and medical expenses. It makes the data enjoy credibility and national representativeness and suitable for our research. Note that limited by the confidentiality agreement of the CLDS dataset, we can only use the CLDS data collected in 2012, 2014, and 2016. In this period, the URRBMI was at the “spontaneous integration” stage. We process the data as follows: (1) Delete individuals participating in the UEBMI or commercial medical insurance and keep the ones only participating in the NCMS, URBMI, or URRBMI. (2) Delete the individuals in cities such as Jiaxing and Dongguan. The NCMS or URBMI in these cities covers both the urban and rural residents at the beginning of its implementation, which means they did not experience the process of integration. (3) Delete the individuals with missing values. In the end, there are 34134 observations in the sample used in this study.

The definitions of the main variables in this study are as follows:

1. *Health*. We use the self-rated health status to measure health. It is a relatively comprehensive and representative indicator, although the self-rated health status may be easily affected by the individual's socioeconomic characteristics and subjective [27]. It is more accurate than objective indicators to some extent [28, 29]. In the CLDS questionnaire, the interviewees were asked “What do you think of your current health?” We define the variable *healthy* based on the question “What do you think of your current health?” in the CLDS questionnaire: *healthy*= 1, if the interviewee answers “very healthy” or “healthy,” and 0 otherwise.
2. *Healthcare*. The “*healthcare*” includes two parts in this article—healthcare utilization and the medical burden that comes along with it. (a) Healthcare utilization. Limited by the data, we describe healthcare utilization by actual use instead of other indicators used by some scholars [30]. Specifically, we construct “*outpatient*” and “*hospital*” variables according to the questions–“whether you went to see a doctor in the past 2 weeks” and “whether you were hospitalized in the past year.” The individual's decision to see a doctor and be hospitalized directly reflects the individual's medical needs and willingness to healthcare utilization. (b) The medical burden. We measure it by the natural logarithms of the out-of-pocket medical expenses of “*outpatient*” and “*hospital*,” which we name “*lnoutself*” and “*lnhosself*.” These self-paid medical expenses reflect the individual's financial burden of healthcare utilization, which can be used to study whether the URRBMI plays a burden-reducing role.
3. *URRBMI*. This is the main explanatory variable in our study. The URRBMI is implemented at the city level or even at the county level, and the city is the smallest administrative unit we can use in the CLDS dataset. Therefore, if the city where the individual's hukou is located has implemented the URRBMI at the survey year, it means the individual is covered by the URRBMI and *URRBMI* = 1; otherwise, *URRBMI* = 0.
4. *Control Variables*. The inequality studied in this article is the socioeconomic inequality in health or healthcare, which means the inequality between people with different socioeconomic status. We measure this socioeconomic difference by income. Considering that there may be endogenous problems in current personal income and current health [31], we use the household income per capita to measure income and take the natural logarithm. Besides, demographic factors such as age, gender, marital status, hukou. and education will affect the individual's health endowment, which affects the individual's decision on healthcare [32, 33]. We also control the year effect and city effect.

### 3.3. Empirical Method

In this article, we use the time-varying DID (difference-in-difference) method to estimate the effects of the URRBMI. Therefore, Equation (3) can be specially written as follows:

(8) $$\begin{array}{c} y_{ict}=\alpha +\beta {\text{URRBMI}}_{ct}+X_{ict}^{\prime }\theta +\mu_{c}+\vartheta_{t}+\varepsilon_{ict}, \end{array}$$

where *β* and *θ* are estimates for the coefficient vector *ρ*_*k*_ in Equation (4). *i* represents the individual, *c* represents the city, and *t* represents the survey year. *y*_*ict*_ is the health or healthcare of individual *i* in year *t*, whose hukou is located in city *c*. URRBMI_*ct*_ varies with city *c* and year *t*, and in the time-varying DID method, it acts as the interaction term of *Treat* and *Time* in traditional DID method. Equation (8) is a regression of *y*_*ict*_ against the URRBMI, a series of control variables (*X*_*ict*_), city fixed effect (*μ*_*c*_) and year fixed effect (*ϑ*_*t*_), and a random error (*ε*_*ict*_).

## 4. Results and Discussion

### 4.1. The Impact of the URRBMI on Health and Healthcare

Table 2 shows the description of the main variables in this study. As it shows, the average coverage rate of the URRBMI is 17.8%, which is in line with the reality at the “spontaneous integration” stage shown in Figure 1.

Columns (1)–(7) in Table 3 list the estimates of the impacts of the URRBMI on health, outpatient utilization, hospital utilization, self-paid outpatient expenses, self-paid hospital expenses, total outpatient expenses, and total hospital expenses. The estimates in columns (1)–(3) show that the URRBMI has a significantly positive effect on health and encourages the utilization of outpatient and hospital at 1% significance level, which to some extent releases individual's medical needs. In columns (4) and (5), it is evident that the URRBMI reduces the self-paid outpatient expenses and self-paid hospital expenses, which eases the individual's medical burden.

### 4.2. Decomposition of the Inequality in Health and Healthcare

We draw the concentration curve of health as shown in Figure 3. It can be seen that the concentration curves of health in 2012–2016 are all below the Fair Line, indicating that there is “pro-rich” health inequality in 2012–2016. Among the concentration curves, the one in 2016 is the lowest, indicating the “size” of the health inequality is the biggest.

However, the role of the URRBMI depends on the decomposition. We calculate the CI to measure health inequality and decompose it based on the estimates in Table 3 column (1). The results are shown in Table 4. From the decomposition results, the CI of health is 0.0963, indicating that there is “pro-rich” health inequality among the insured. It is consistent with the conclusion we get from Figure 3, that is compared with the low-income groups, the high-income groups enjoy health advantages. The contribution rate of the URRBMI to health inequality is 0.84%, with a contribution of 0.0008, which suggests that the URRBMI promotes the expansion of health inequality. Specific to the two components of the URRBMI's contribution, both the CI and the elasticity are positive. The positive CI indicates that the implementation of the URRBMI favors the high-income groups. That is, the high-income groups are more likely to be insured. Moreover, the positive elasticity reflects that the URRBMI has a positive direct impact on health. The CI is greater than the elasticity, meaning that the CI, or the inequality of the URRBMI, plays a major role in its contribution.

By comparing the contributions of different variables, it is evident that factors such as income and age play a dominant role in producing health inequality. The primary source of their contribution is elasticity, suggesting that their direct impact on health mainly causes health inequality. While the contribution of secondary education mainly comes from its inequality, which indicates that the inequality in secondary education dominates its contribution to health inequality. The contribution of URRBMI only accounts for 1.66% of income and 16.25% of secondary education. Compared with these factors, although the URRBMI does contribute to health inequality, it is much smaller.

Taking outpatient as an example, we draw the concentration curve of healthcare in Figure 4. We can see that the concentration curves of outpatient in 2012–2016 are all above the Fair Line, which means that the inequality in 2012–2016 is “pro-poor.” The concentration curve in 2014 is the lowest, indicating the “size” of inequality in outpatient utilization is the smallest.

We also decompose the inequality in healthcare, and the results are shown in Table 5—only the part of the URRBMI demonstrated. In Panel *A* and Panel *B*, the CIs of outpatient and hospital are negative, reflecting inequality in healthcare utilization in favor of the low-income groups. The CIs of lnoutself and lnhosself in Panel *C* and Panel *D* are positive, indicating that the low-income groups enjoy relatively low out-of-pocket medical expenses and light medical burden. Therefore, both the healthcare utilization and the burden of medical expenses are beneficial to the low-income groups, the same as the concentration curve shown in Figure 4.

Note that the contribution rates of the URRBMI in all the panels are negative, which means that the URRBMI eases the inequality between different income groups. The CI of the URRBMI is positive, and its absolute value is greater than elasticity, the same as the decomposition result of health inequality. It indicates that both in the inequality in health and healthcare, the contribution of the URRBMI mainly comes from its own “pro-rich” inequality.

### 4.3. Decomposition of Inequality between Groups

It can be seen from the above analysis that the URRBMI plays different roles in the inequality in health and healthcare. We are curious about how it contributes to the inequality in different areas and regions (intragroup), especially between areas and regions (intergroup). Therefore, we further divide the inequality in health and healthcare into intragroup inequality and intergroup inequality. The results are shown in Table 6.

According to Table 6 Panel *A*, the health's CIs of urban, rural, east, and non-east are 0.0866, 0.0946, 0.0807, and 0.0959, respectively, which indicates that they all have “pro-rich” health inequality of different “sizes,” and the “size” is even greater in the rural areas and non-east regions. Besides, the health's CI between the urban and rural areas is 0.0026, which means that the urban residents take the health advantages. And the health's CI between the east and non-east regions is 0.0058, indicating that residents in the east take the health advantages. In Table 6 Panel *B*, the intragroup CIs of healthcare utilization are negative and the intragroup CIs of medical burden are positive. It suggests that intragroup inequalities in areas and regions are all “pro-poor” and the healthcare utilization medical burden benefit the low-income groups. Besides, the intergroup CIs of outpatient and hospital are positive and the intergroup CIs of lnhosself are negative, meaning the inequalities between areas and regions are “pro-rural” and “pro-non-east.” While the intergroup CIs of lnoutself are negative, the inequalities are “pro-urban” and “pro-east.”

In China, the rural areas and the non-east regions are underdeveloped. Broadly speaking, both the intragroup health inequality and the intergroup health inequality are inclined to the economically developed areas, regions, and groups. In contrast, those of the healthcare are inclined to the economically backward ones.

The URRBMI demonstrates the same inclination as the health inequality—it favors the economically affluent areas, regions, and groups. Its contribution rates to health are positive, indicating that it enlarges the health inequality. However, its contribution rates to the intergroup healthcare inequality are almost all negative, which suggests that to some extent, the URRBMI narrows the gap in healthcare between areas and regions.

### 4.4. Changes of the Inequality and the URRBMI's Contribution

To better study the changes in health and healthcare inequality and figure out the dominant part of the URRBMI in its contribution, we calculate the CIs in 2012, 2014, and 2016, and decompose the contribution of the URRBMI.

Table 7 reports the CIs of health and healthcare in 2012, 2014, and 2016. In Panel *A*, we can see that the CIs of health in 2012, 2014, and 2016 are 0.1068, 0.076, and 0.1064, respectively. Although the “size” of inequality in 2014 shows a relatively small and brief decline, we can still find health inequality in favor of the high-income groups in each year. The CIs of the URRBMI are positive in 2012, 2014, and 2016, and it has increased dramatically. It reveals that the favorable populations who are more likely and easily covered by the URRBMI are always the high-income groups, and the coverage inequality increases along the time. It deserves to be mentioned that the contribution rates of the URRBMI are −0.05%, 0.7%, and 1.86% in 2012, 2014, and 2016, respectively. Although the URRBMI alleviated the health inequality in 2012, it turned to the opposite side to breed health inequality in 2014, with its contribution increasing with time.

From Table 7 Panel *B*–Panel *E*, the CIs of outpatient and hospital are all negative, and the CIs of lnoutself and lnhosself are almost all positive, with the absolute values showing an escalating trend overall. We can infer that both the healthcare utilization and the medical burden benefit the low-income groups with an expansion of the inequality. As shown in Table 7 column (6), on the whole, the contribution rates of the URRBMI to the inequality in healthcare are on the decline, showing a decreasing contribution of the URRBMI to the healthcare inequality.

Table 8 reports the changes and decompositions of the URRBMI's contributions. We decompose the change of the URRBMI's contribution into CI's change and elasticity's change to clarify which plays the dominant role.

Table 8 shows that the change of the URRBMI's contribution to inequality within the three periods is mainly derived from its elasticity's change. Taking health as an example, Table 7 Panel *A* shows that the CI of the URRBMI increases from 0.0369 to 0.1346 from 2012 to 2016, reflecting a deepening “pro-rich” inequality in coverage. Meanwhile, the URRBMI's elasticity jumps from −0.0016 to 0.0147, which indicates that 1% increase in the coverage of the URRBMI will bring about 0.0147% health inequality. It will undoubtedly worsen the situation for the low-income groups, where they have to face a “dual-disadvantage” in terms of coverage and health.

In summary, there is “pro-rich” inequality in health, and the URRBMI's contribution to it is increasing year by year. Also, there is “pro-poor” inequality in healthcare, and the URRBMI's contribution to it is declining on the whole. Although the URRBMI has a growing “pro-rich” inequality itself, the elasticity's change dominates the change of its contribution to the inequality in health and healthcare.

### 4.5. Heterogeneity

Before this section, the study and discussion on inequality suggest that the URRBMI reduces the “pro-poor” healthcare inequality but exacerbates the “pro-rich” health inequality. Meanwhile, the economic intuition and many literature studies generally believe that people with lower incomes are often more sensitive to the price of healthcare. So medical insurance can improve their access to healthcare, which directly affects health [34]. Therefore, we propose the hypothesis: the URRBMI's promotion effect in health and healthcare is mainly reflected in the low-income groups. We divide the sample into quarters according to the income to study underlying heterogeneity and the results are shown in Table 9.

According to the results, the URRBMI significantly promotes outpatient and hospital utilization by the top 50% and top 75% of the low-income people, with the lower-income groups benefiting more. Besides, the URRBMI reduces the self-paid outpatient and hospital expenses, with the lower-income groups benefiting more similarly. In terms of health, both the health status of the lowest-income group and the highest-income group get improved. We can find that against the existence of “pro-rich” health inequality, the growing use of medical resources encouraged by the “pro-poor” healthcare inequality does help to improve the health of the lowest-income groups. Therefore, the lowest-income groups benefit the most from the URRBMI.

We attempt to explain the seemingly contradictory conclusion that “pro-poor” healthcare inequality coexists with “pro-rich” health inequality. Generally speaking, the “pro-poor” healthcare inequality should cause “pro-poor” health inequality. However, due to the fragmented operation of the Basic Medical Insurance, there are huge gaps in the health stocks of people in different areas, regions, and groups [35]. Although the residents, especially those with low income, are encouraged to use medical services by the URRBMI and the “pro-poor” healthcare inequality, the existing disparity in health stock still allows the high-income groups to enjoy a health advantage. Therefore, although the URRBMI may have an incremental effect for the vertical comparison of the individual's health, for the horizontal comparison of health between people of different groups, it fails to alleviate the existed health gap.

### 4.6. Robustness Check

This study uses the time-varying DID method to estimate the impact of the URRBMI on health and healthcare. The regression results are the basis of the subsequent decomposition of the concentration index and discussion about inequality. Therefore, the credibility of the conclusions depends on the credibility of the regression results, and we conduct two robustness tests.

#### 4.6.1. PSM-DID (Difference-In-Difference Based on the Propensity Score Matching)

Considering the endogeneity problem caused by selection bias and the possible systemic differences between the insured group and their counterparts, we use the PSM-DID method to estimate the impact of the URRBMI again. By selecting the insured and its “counterfactual” control group from the common support domain, the PSM-DID method ensures their homogeneity and comparability. The results are shown in Table 10. The estimated results are consistent with those in Table 3, which means the results of this study are relatively robust.

#### 4.6.2. Placebo Test

For possible non-randomization caused by the influence of other factors that may exist, we conduct a placebo test by constructing a random falsification treated group. Specifically, we randomly select individuals as insured and repeat the previous regression 500 times.  Figure 5 shows the 500 regression results for health and healthcare. The curve is the kernel probability density distribution of the estimates, and the vertical dashed line is the estimated coefficients in Table 3.

Figure 5 shows that the estimates of 500 regressions are mainly concentrated near 0, which is quite different from the estimated coefficients. Therefore, we can infer that the results in this study are unlikely to be accidental events and are relatively robust.

## 5. Conclusion

In the context of the fragmented operation of China's Basic Medical Insurance, the gap between areas, regions, and groups in health and healthcare cannot be ignored. Under this situation, the URRBMI has been implemented in China. Whether to reduce inequality and promote fairness is a crucial indicator for evaluating the integrating reform, that is, the URRBMI.

This study uses the time-varying DID method and decomposes the concentration index based on the CLDS data in 2012, 2014, and 2016 to examine the role of the URRBMI in health and healthcare inequality. The results show that: (1) There is a “pro-rich” coverage inequality in the URRBMI with an increasing trend. (2) The URRBMI significantly improves health, but expands health inequality among different income groups, with its contribution growing year by year. (3) The URRBMI evidently promotes healthcare utilization, reduces the medical burden, and narrows the gap among different income groups, although this effect is generally on a downward trend. In addition, the decomposition of inequality in health and healthcare between areas and regions also shows roughly the same result: the URRBMI enlarges the health inequality but reduces the healthcare inequality between the urban and rural areas and between the east and non-east regions. What's more, although the URRBMI demonstrates a seemingly contradictory effect on the inequality in health and healthcare, it favors the lowest-income group the most. In summary, the implementation of the URRBMI has achieved some phased results, but it is still insufficient in alleviating health inequality. As mentioned above, the gap in the health stock of people in different groups has a long history, which is caused mainly by the misallocation of medical resources between areas and regions and may further deepen health inequality. In addition, the URRBMI itself is “pro-rich,” which goes against the original intention of “integrating.”

These findings can provide policy implications for policymakers. In the follow-up practice of the URRBMI, the coverage, drug list, and healthcare providers deserve more attention to benefit people insured and reduce inequality. Specifically, to ensure that individuals have equal access to medical services, the central government and local governments should increase their investment in medical resources, especially in economically underdeveloped areas and regions. Constructing the hierarchical medical system and medical treatment combination is an excellent way to balance the distribution of medical resources between areas and regions. In addition, considering the social insurance nature of the URRBMI, its coverage should be moderately inclined to the low-income groups, thereby reducing their worries and encouraging timely healthcare utilization.

There is a limitation of our research that needs to be acknowledged. Due to the confidentiality agreement of the CLDS, the variable URRBMI can only be defined by the city's implementation rather than the county's implementation. It may limit the regression results in this study to some extent. This is left to us or researchers interested to further perfect this study with more detailed data.

## Figures and Tables

**Figure 1:** The number of participants in the URRBMI.

**Figure 2:** Concentration curve.

**Figure 3:** The concentration curve of health.

**Figure 4:** The concentration curve of outpatient.

**Figure 5:** Placebo test.

**Table 1:** Notations and definitions.

Notations	Definitions
CI	Concentration index. It measures the inequality.
CI(*y|I*)	The CI of *y* (health or healthcare).
CI(*x*_*k*_*|I*)	The CI of influencing factor *x*_*k*_.
*η*_*k*_	The elasticity of *y* to *x*_*k*_.
*η*_*k*_ CI(*x*_*k*_*|I*)	*x*_*k*_'s contribution
CI_*u*_(*y|I*)	The intragroup inequality of urban residents
CI_*r*_(*y|I*)	The intragroup inequality of rural residents
CI_*ur*_(*y|I*)	The intergroup inequality of urban and rural residents
CI_*e*_(*y|I*)	The intragroup inequality of the east region
CI_*ne*_(*y|I*)	The intragroup inequality of the non-east region
CI_*b*_(*y|I*)	The intergroup inequality of the east region and the non-east region
ΔCI(*y|I*)	The change of *y*'s CI from period *t* − 1 to *t*
ΔCI(*x*_*k*_*|I*)	The change of *x*_*k*_'s CI from period *t* − 1 to *t*
Δ*η*_*k*_	The change of *y*'s elasticity to *x*_*k*_ from period *t* − 1 to *t*
CI_*t*_(*x*_*k*_*|I*)	*x*_*k*_'s CI in period *t*
*η*_*kt*_	*y*'s elasticity to *x*_*k*_ in period *t*

**Table 2:** Description of main variables.

Variables	Meaning	N	Mean	Sd.
Healthy	Self-rated health status: healthy = 1; 0 otherwise	34134	0.557	0.497
Outpatient	If the individual went to see a doctor in the past 2 weeks: outpatient = 1; 0 otherwise	34134	0.087	0.281
Hospital	If the individual was hospitalized in the past year: hospital = 1; 0 otherwise	34134	0.081	0.273
Lnoutexp	Natural logarithm of the deflated total outpatient expenses in the past 2 weeks	2979	5.598	2.256
Lnhosexp	Natural logarithm of the deflated total hospitalization expenses in the past year	2797	8.415	1.564
Lnoutself	Natural logarithm of the deflated self-paid outpatient expenses in the past 2 weeks	2979	4.246	2.844
Lnhosself	Natural logarithm of the deflated self-paid hospitalization expenses in the past year	2797	6.836	2.936
URRBMI	If the individual is insured by the URRBMI: URRBMI = 1; 0 otherwise	34134	0.178	0.383
Lnpcincome	Natural logarithm of the deflated household income per capita	34134	8.642	1.593
Male	Male = 1; 0 otherwise	34134	0.473	0.499
Age	Age	34134	45.590	14.560
Rural	If the individual's hukou is located in the rural areas, rural = 1; 0 otherwise,	34134	0.890	0.313
Married	Married = 1; 0 otherwise	34134	0.831	0.374
Illit	Did not receive formal education = 1; 0 otherwise	34134	0.171	0.376
Priedu	Primary education = 1; 0 otherwise	34134	0.628	0.483
Secedu	Secondary education = 1; 0 otherwise	34134	0.124	0.329
Highedu	Bachelor or college degree = 1; 0 otherwise	34134	0.037	0.189
Superhigh	Master or doctor degree = 1; 0 otherwise	34134	0.001	0.026
Pension	If the individual has a pension: pension = 1; 0 otherwise	34134	0.521	0.500
Hhnum	Family size	34134	3.961	1.819
Sanitary	If the house has tap water or indoor toilet: sanitary = 1; 0 otherwise	34134	0.849	0.358
East	If the province where the individual's hukou is located in belongs to the east region: east = 1; 0 otherwise	34134	0.353	0.478

“N” refers to the number of observations used; “Sd.” refers to standard deviation.

**Table 3:** The impact of the URRBMI on health and healthcare.

Variables	(1)	(2)	(3)	(4)	(5)
	Healthy	Outpatient	Hospital	Lnoutself	Lnhosself
URRBMI	0.0243^*∗∗∗*^ (0.0068)	0.0246^*∗∗∗*^ (0.0085)	0.0278^*∗∗∗*^ (0.0082)	−1.0740^*∗∗∗*^ (0.1363)	−0.4289^*∗∗∗*^ (0.1646)
Age	−0.0210^*∗∗∗*^ (0.0012)	0.0039^*∗∗∗*^ (0.0007)	−0.0013^*∗*^ (0.0007)	0.0266 (0.0238)	0.0502^*∗∗*^ (0.0250)
Age2	0.0001^*∗∗∗*^ (0.0000)	−0.0000^*∗∗∗*^ (0.0000)	0.0000^*∗∗∗*^ (0.0000)	−0.0005^*∗∗*^ (0.0003)	−0.0007^*∗∗*^ (0.0003)
Male	0.0606^*∗∗∗*^ (0.0052)	−0.0268^*∗∗∗*^ (0.0031)	−0.0214^*∗∗∗*^ (0.0031)	0.3602^*∗∗∗*^ (0.1061)	0.2829^*∗∗*^ (0.1179)
Marriage	0.0685^*∗∗∗*^ (0.0088)	−0.0212^*∗∗∗*^ (0.0053)	0.0126^*∗∗*^ (0.0052)	0.3321^*∗*^ (0.1700)	0.1025 (0.1875)
Hhnum	0.0012 (0.0014)	0.0007 (0.0009)	0.0000 (0.0009)	−0.2950^*∗∗∗*^ (0.0281)	−0.1597^*∗∗∗*^ (0.0300)
Lnpcincome	0.0367^*∗∗∗*^ (0.0017)	−0.0058^*∗∗∗*^ (0.0010)	−0.0072^*∗∗∗*^ (0.0010)	0.0433 (0.0305)	0.0752^*∗∗*^ (0.0312)
Rural	0.0135 (0.0086)	0.0051 (0.0059)	−0.0024 (0.0058)	0.0128 (0.1889)	−0.5041^*∗∗*^ (0.1988)
Priedu	0.0672^*∗∗∗*^ (0.0068)	−0.0174^*∗∗∗*^ (0.0043)	−0.0095^*∗∗*^ (0.0042)	−0.6758^*∗∗∗*^ (0.1176)	−0.1403 (0.1332)
Secedu	0.1224^*∗∗∗*^ (0.0100)	−0.0293^*∗∗∗*^ (0.0062)	−0.0126^*∗∗*^ (0.0061)	−0.6956^*∗∗∗*^ (0.2161)	−0.6857^*∗∗∗*^ (0.2297)
Highedu	0.1684^*∗∗∗*^ (0.0157)	−0.0276^*∗∗∗*^ (0.0096)	−0.0147 (0.0095)	−0.8669^*∗*^ (0.4451)	−0.3383 (0.4753)
Superhigh	0.3003^*∗∗∗*^ (0.0957)	0.0194 (0.0564)	−0.0122 (0.0557)	1.8758 (1.9297)	−0.2324 (2.9103)
Pension	0.0229^*∗∗∗*^ (0.0053)	0.0038 (0.0034)	0.0034 (0.0033)	−0.1324 (0.1055)	−0.0194 (0.1153)
Sanitary	0.0205^*∗∗∗*^ (0.0072)	−0.0106^*∗∗*^ (0.0050)	−0.0027 (0.0049)	−0.3828^*∗∗∗*^ (0.1361)	−0.3301^*∗∗*^ (0.1466)
Constant	0.6973^*∗∗∗*^ (0.0299)	0.1139^*∗∗∗*^ (0.0343)	0.1365^*∗∗∗*^ (0.0327)	5.6156^*∗∗∗*^ (0.6186)	6.8977^*∗∗∗*^ (0.6641)
Year effect	Controlled	Controlled	Controlled	Controlled	Controlled
City effect	Controlled	Controlled	Controlled	Controlled	Controlled
Observations	34,134	34,134	34,134	2,979	2,797
R-squared	0.1179	0.0645	0.0351	0.0912	0.0296

Standard errors in parentheses, ^*∗∗∗*^*p* < 0.01, ^*∗∗*^*p* < 0.05, and ^*∗*^*p* < 0.1.

**Table 4:** Decomposition of health inequality.

Variables	(1)	(2)	(3)	(4)	(5)	(6)
	Coefficient ${\hat{\rho }}_{k}$	Mean ${\bar{x}}_{k}$	Elasticity *η*_*k*_	Concentration index *CI*(*x*_*k*_*|I*)	Contribution	Contribution rate (%)
Healthy		0.557		0.0963		
URRBMI	0.0243	0.1783	0.0077	0.1042	0.0008	0.84
Age	−0.0210	45.59	−1.7191	−0.0193	0.0332	34.48
Age2	0.0001	2290	0.5393	0.0399	−0.0215	−22.36
Male	0.0606	0.473	0.0515	−0.0046	−0.0002	−0.25
Marriage	0.0685	0.831	0.1023	−0.0013	−0.0001	−0.14
Hhnum	0.0012	3.960	0.0084	−0.0650	−0.0005	−0.57
Lnpcincome	0.0367	8.642	0.5696	0.0858	0.0489	50.75
Rural	0.0135	0.890	0.0215	−0.0403	−0.0009	0.90
Priedu	0.0672	0.628	0.0759	−0.0014	−0.0001	0.11
Secedu	0.1224	0.124	0.0271	0.1834	0.0050	5.17
Highedu	0.1684	0.037	0.0112	0.3939	0.0044	4.57
Superhigh	0.3003	0.001	0.0004	0.5777	0.0002	0.23
Pension	0.0229	0.521	0.0214	−0.0063	−0.0001	−0.14
Sanitary	0.0205	0.849	0.0312	0.0356	0.0011	1.15

**Table 5:** Decomposition of the inequality in healthcare.

Variables	(1)	(2)	(3)	(4)	(5)	(6)
	Coefficient ${\hat{\rho }}_{k}$	Mean ${\bar{x}}_{k}$	Elasticity *η*_*k*_	Concentration index CI(*x*_*k*_*|I*)	Contribution	Contribution rate (%)
*A: outpatient*						
Outpatient		0.0866		−0.1064		
URRBMI	0.0246	0.1783	0.0506	0.1041	0.0053	−4.95

*B: hospital*						
Hospital		0.0814		−0.1114		
URRBMI	0.0278	0.1783	0.0610	0.1041	0.0064	−5.71

*C: lnoutself*						
Lnoutself		4.2460		0.0186		
URRBMI	−1.0740	0.1722	−0.0436	0.0899	−0.0039	−21.08

*D: lnhosself*						
Lnhosself		6.8361		0.0206		
URRBMI	−0.4289	0.1334	−0.0084	0.1371	−0.0011	−5.58

**Table 6:** Decomposition of inequality between groups.

	*N*	Total CI	CI of the URRBMI	Contribution rate (%)
*A: health*				

*Healthy*	34134	0.0963	0.1042	0.84

Subsample: Urban and rural				
Urban	3759	0.0866	0.0646	0.43
Rural	30375	0.0946	0.0889	0.77
Between		0.0026	0.0180	0.11

Subsample: East and non-east				
East	12049	0.0807	−0.0204	0.82
Non-east	22085	0.0959	0.1733	0.58
Between		0.0058	−0.0007	0.18

*B: healthcare*				

*Outpatient*	34134	−0.1064	0.1042	−4.95

Subsample: Urban and rural				
Urban	3759	−0.0745	0.0646	−10.21
Rural	30375	−0.1027	0.0889	−3.85
Between		−0.0068	0.0180	−0.40

Subsample: East and non-east				
East	12049	−0.0324	−0.0204	3.54
Non-east	22085	−0.1012	0.1733	−2.80
Between		−0.0295	−0.0007	−4.39

*Hospital*	34134	−0.1114	0.1042	−5.71

Subsample: Urban and rural				
Urban	3759	−0.0978	0.0646	3.24
Rural	30375	−0.1065	0.0889	−6.32
Between		−0.0059	0.0180	−0.44

Subsample: East and non-east				
East	12049	−0.0181	−0.0204	7.60
Non-east	22085	−0.1169	0.1733	−3.34
Between		−0.0294	−0.0007	−6.23

*Lnoutself*	2979	0.0186	0.0889	−21.08

Subsample: Urban and rural				
Urban	254	0.0108	0.1611	−115.37
Rural	2725	0.0218	0.0549	−10.32
Between		−0.0023	0.0250	−1.80

Subsample: East and non-east				
East	895	0.0391	−0.0251	11.62
Non-east	2084	0.0120	0.1289	−9.19
Between		−0.0015	0.0063	−18.14

*Lnhosself*	2797	0.0206	0.1371	−5.58

Subsample: Urban and rural				
Urban	264	−0.0162	0.2397	8.66
Rural	2533	0.0236	0.1082	−3.96
Between		0.0008	0.0165	−2.81

Subsample: East and non-east				
East	769	0.0243	−0.0116	1.27
Non-east	2028	0.0154	0.1413	−8.29
Between		0.0028	0.0378	0.08

**Table 7:** The CIs in 2012–2016.

Year	Total CI	*N*	URRBMI					
			(1)	(2)	(3)	(4)	(5)	(6)
			Coefficient ${\hat{\rho }}_{k}$	Mean ${\bar{x}}_{k}$	Elasticity *η*_*k*_	CI(*x*_*k*_*|I*)	Contribution	Contribution rate (%)
*A: healthy*								
2012	0.1068	9102	−0.0083	0.0985	−0.0016	0.0369	−0.0001	−0.05
2014	0.0760	13020	0.0155	0.1479	0.0039	0.1369	0.0005	0.70
2016	0.1064	12012	0.0301	0.2717	0.0147	0.1346	0.0020	1.86

*B: outpatient*								
2012	−0.1243	9102	0.9998	0.0985	0.5995	0.0369	0.0217	−17.48
2014	−0.0657	13020	−0.0126	0.1479	−0.0360	0.1369	−0.0049	7.40
2016	−0.1199	12012	−0.0026	0.2717	−0.0108	0.1346	−0.0015	1.22

*C: hospital*								
2012	−0.0802	9102	−0.0501	0.0985	−0.0475	0.0369	−0.0017	2.11
2014	−0.1125	13020	0.9104	0.1479	2.0557	0.1369	0.2796	−248.59
2016	−0.1331	12012	−0.0055	0.2717	−0.0184	0.1346	−0.0025	1.86

*D: lnoutself*								
2012	0.0050	1495	−1.0168	0.0977	−0.0183	0.0663	−0.0012	−23.95
2014	−0.0003	684	−0.6756	0.2295	−0.0324	0.1212	−0.0039	1549.17
2016	0.0103	800	−0.1146	0.2625	−0.0191	0.0840	−0.0016	−15.66

*E: lnhosself*								
2012	0.0098	946	0.7719	0.0423	0.0042	0.0789	0.0003	3.38
2014	0.0116	861	0.2934	0.1034	0.0042	0.2052	0.0009	7.41
2016	0.0234	990	0.0552	0.2465	0.0024	0.1632	0.0004	1.70

**Table 8:** Changes and decompositions of contributions.

Period	The total contribution of the URRBMI	Contribution of CI's change *η*ΔCI	Contribution of elasticity's change CIΔ*η*
*A: healthy*			
2012–2014	0.0006	−0.0002	0.0008
2014–2016	0.0015	−0.0000	0.0015
2012–2016	0.0021	−0.0001	0.0022

*B: outpatient*			
2012–2014	−0.0266	0.0599	−0.0865
2014–2016	0.0034	0.0001	0.0033
2012–2016	−0.0232	0.0588	−0.0820

*C: hospital*			
2012–2014	0.2813	−0.0048	0.2861
2014–2016	−0.2821	−0.0030	−0.2792
2012–2016	−0.0008	−0.0047	0.0039

*D: lnoutself*			
2012–2014	−0.0027	−0.0010	−0.0017
2014–2016	0.0023	0.0012	0.0011
2012–2016	−0.0004	−0.0004	−0.0000

*E: lnhosself*			
2012–2014	0.0006	0.0005	0.0001
2014–2016	−0.0005	−0.0002	−0.0003
2012–2016	0.0001	0.0003	−0.0002

**Table 9:** Heterogeneity analysis of different income groups.

Variables	Lowest-income groups	Lower-income groups	Higher-income groups	Highest-income groups
Healthy	0.0297^*∗∗*^ (0.0150)	0.0035 (0.0139)	0.0042 (0.0133)	0.0283^*∗∗*^ (0.0123)
Outpatient	0.0551^*∗∗*^ (0.0229)	0.0519^*∗∗∗*^ (0.0185)	0.0081 (0.0156)	0.0080 (0.0139)
Hospital	0.0519^*∗∗*^ (0.0231)	0.0356^*∗∗*^ (0.0174)	0.0327^*∗∗*^ (0.0151)	0.0046 (0.0134)
Lnoutself	−1.2448^*∗∗∗*^ (0.2568)	−1.1639^*∗∗∗*^ (0.2587)	−1.1682^*∗∗∗*^ (0.2869)	−0.5463^*∗*^ (0.2996)
Lnhosself	−0.7299^*∗∗*^ (0.3154)	−0.6712^*∗∗*^ (0.3367)	−0.2882 (0.3254)	0.0460 (0.3445)
Control variables	Yes	Yes	Yes	Yes
Year effect	Controlled	Controlled	Controlled	Controlled
City effect	Controlled	Controlled	Controlled	Controlled
Observations	8698	8601	8453	8382

**Table 10:** The estimates of PSM-DID.

Variables	Healthy	Outpatient	Hospital	Lnoutself	Lnhosself
URRBMI	0.0242^*∗∗∗*^ (0.0068)	0.0238^*∗∗∗*^ (0.0085)	0.0270^*∗∗∗*^ (0.0082)	−1.0724^*∗∗∗*^ (0.1367)	−0.4314^*∗∗∗*^ (0.1654)
Constant	0.6973^*∗∗∗*^ (0.0299)	0.1139^*∗∗∗*^ (0.0343)	0.1365^*∗∗∗*^ (0.0327)	5.6156^*∗∗∗*^ (0.6186)	6.8977^*∗∗∗*^ (0.6641)
Control variables	Yes	Yes	Yes	Yes	Yes
Year effect	Controlled	Controlled	Controlled	Controlled	Controlled
City effect	Controlled	Controlled	Controlled	Controlled	Controlled
Observations	33,890	33,890	33,890	2,936	2,762
*R*-squared	0.1179	0.0639	0.0345	0.0905	0.0290

## Data Availability

The data used in this study are derived from the China Labor-force Dynamic Study (CLDS). The data are open to people who have registered and submitted their applications. Data are available at http://css.sysu.edu.cn/. People can also apply for the data by sending application emails to cssdata@mail.sysu.edu.cn.
